The article "Experimental Study on the Central Mechanism of Penehyclidine Hydrochloride against Relapse Behavior in Morphine-Dependent Rats" was retracted in 2023. Reasons: signs of a paper mill; suspected computer-generated content; unreliable results or conclusions; concerns about the data.

# Experimental Study on the Central Mechanism of Penehyclidine Hydrochloride against Relapse Behavior in Morphine-Dependent Rats

**DOI:** 10.1155/2022/7785714

**Published:** 2022-01-27

**Authors:** Yufeng Zou, Zhe Jin, Meng Yun Li, Lijuan Tang, Kai Chen

**Affiliations:** Department of Anesthesiology, Zhongnan Hospital of Wuhan University, Wuhan, 430071 Hubei, China

## Abstract

**Objective:**

This article is mainly to study the central mechanism of penehyclidine hydrochloride against relapse behavior in morphine-dependent rats.

**Methods:**

The rats were randomly divided into the blank control group (k), PHC low-dose group (LP according to a body weight of 0.22 mg/kg), middle-dose group (MP according to a body weight of 0.55 mg/kg), high-dose group (HP according to a body weight of 1.38 mg/kg), and administration group, with 40 rats in each group. Each group was randomly divided into 5 subgroups (*n* = 10): 4 h after administration, 7 h after administration, 13 h after administration, 25 h after administration (K48, LP48, MP48, and HP48), and 37 h after administration, and then, Morris water maze experiment and immunohistochemical detection of the rat brain hippocampus were carried out.

**Results:**

4 and 7 hours after administration, compared with group 1, the TchE activity increased and Ach level decreased in groups 2, 3, and 4 and the difference was significant (*P* < 0.05), so the principle of penehyclidine hydrochloride against morphine-dependent rats is that penehyclidine hydrochloride causes cognitive impairment in the brain of mice, thereby achieving antimorphine effects.

## 1. Introductions

In recent years, neuroscience and behavioral science research of drug addiction have made many progress [1, 2]. Although its complex mechanism of action is not yet clear, many studies have shown that drug addiction is a chronic and recurrent encephalopathy and its root cause is addictive memory [3, 4]. A large number of studies have confirmed that the central and peripheral cholinergic nervous systems play an important role in the production of morphine dependence. Cholinergic drugs can exacerbate opioid withdrawal symptoms, and muscarinic and nicotinic inhibitors can relieve some withdrawal symptoms [5, 6]. In clinical practice, scopolamine M receptor antagonists have also shown significant effects in relieving withdrawal symptoms. Phencyclidine hydrochloride (PHC) is a new type of selective anticholinergic drug with central sedative effect. Although it is widely used clinically as a preoperative drug, there is no experimental research report on its use in morphine addiction [7, 8]. Drug dependence refers to the characteristics that drugs interact with the body for a long time, resulting in specific, compensatory, and adaptive changes in physiological function, biochemical process, and/or morphology. Stopping medication can lead to discomfort and/or psychological desire. Drug dependence is a mental state caused by the interaction between drugs and the body, sometimes including the physical state, showing a compulsive behavior and other reactions to use the drug continuously or regularly.

For antimorphine dependence research, some researchers are currently studying effective drugs for the treatment of psychological addiction caused by opioids, but because the addiction mechanism is not fully understood and the symptoms are complex, single-target drugs cannot solve it. Foreign Western medicine also has no good strategy to solve this problem [9]. Some researchers have proposed that in our country's long-term medication practice, traditional Chinese medicine can improve the desire, pain, and general discomfort caused by multiple links, multiple uses, and multiple systems and some research results have been made in this regard and preliminary research is ongoing. Traditional herbal detoxification has a positive effect on controlling withdrawal symptoms, prolonging symptoms and preventing recurrence. Nowadays, typical traditional detoxification Chinese medicines, such as Wei'an Huisheng Oral Liquid, Huishengkang, Humen Mixture, and Baokang Jiedu Granules, can effectively alleviate the drug-induced of withdrawal symptoms. For example, Yi'an Huisheng Oral Liquid can reconcile qi and blood, warm the spleen, and nourish the kidney. Ginseng has the effects of detoxification, soothing the nerves, nourishing the kidney, and nourishing the liver, which can reduce the detoxification time and side effects. Baogan Jiedu granules have a sedative effect, and this drug may reduce the effectiveness of withdrawal symptoms. In addition, acupuncture is widely used as a traditional medical treatment in our country to help eliminate drug addiction. Studies have shown that heroin-dependent patients can effectively reduce withdrawal symptoms with the help of acupuncture [10]. Some researchers have proposed that PHC is a new class of drugs that can interact with cholinergic receptors (M receptors) independently developed by our country. It is an anticholinergic drug and has strong central and peripheral anticholinergic drugs [11]. In summary, there are many research results on antimorphine dependence and penehyclidine hydrochloride, but relatively few studies on antimorphine dependence and penehyclidine hydrochloride. Targeted drugs refer to drugs or their preparations endowed with targeting ability. The purpose is to make the drug or its carrier aim at the specific lesion site and accumulate or release-effective components at the target site. The targeted preparation can make the drug form a relatively high concentration in the target part, so as to improve the efficacy, inhibit the toxic and side effects, and reduce the damage to normal tissues and cells.

This article studies the central mechanism of penehyclidine hydrochloride against the relapse behavior of morphine-dependent rats. Based on relevant literature data, the mechanism of morphine addiction, penehyclidine hydrochloride against morphine, and the central mechanism related to the addiction mechanism, the analysis was carried out separately, and then, the central mechanism experiment of penehyclidine hydrochloride against the relapse behavior of morphine-dependent rats was carried out and relevant conclusions were drawn through the experiment. Its derivative morphine hydrochloride is a commonly used anesthetic in clinics. It has strong analgesic effect. It is mostly used for severe pain caused by trauma, operation, and burn. It is also used for angina pectoris caused by myocardial infarction. It can also be used as analgesic, antitussive, and antidiarrheal agents. The diacetate of morphine is also known as heroin. But its biggest disadvantage is addiction. This makes long-term smokers have a serious dependence on morphine both physically and psychologically, resulting in serious toxicosis, which does great harm to themselves and the society.

## 2. Study on Penehyclidine Hydrochloride and Antimorphine Dependence

### 2.1. The Mechanism of Morphine Addiction

The process of morphine addiction is essentially a series of adaptive changes that occur after the body is stimulated by exogenous morphine for a long time. This change occurs at the tissue, cell, and molecular level. When the drug is stopped suddenly, the body becomes steady and there are many withdrawal symptoms. Some people think that after long-term use of opioids, the body is particularly sensitive to drugs. This high sensitivity is usually latent. When the drug is withdrawn, this hypersensitivity reaction will be manifested in a state of excitement such as recovery, which will cause withdrawal symptoms. Others believe that the causes of addiction include positive reinforcement and negative reinforcement. Positive reinforcement refers to the psychological stimulation caused by the use of substances such as rewards and euphoria, while negative reinforcement refers to a series of withdrawals. These physical symptoms include nervous system damage, appearance, and memory loss.

Studies have shown that DA neural pathways are related to morphine addiction [12]. DA is an important messenger of the reward mechanism in the brain and participates in the formation of drug-seeking behavior and euphoria. The application of exogenous opioids will increase the dopamine content in the nucleus accumbens, promote the release of endogenous opioid peptides in GABA neurons, reduce the GABA content in the abdominal bulb, ultimately weaken the inhibition of DA neurons, promote DA release, and cause addiction symptoms and intracranial adaptability. After morphine withdrawal symptoms cease, DA release increases, DA cell response increases, and withdrawal symptoms appear. Morphine withdrawal symptoms block Ca2+ channels and prevent Ca2+ influx, intracellular Ca2+ decreases, and Ach decreases. Ach is a major neurotransmitter, which is closely related to learning, memory, and memory impairment. Generally, Ca 2+ is required to participate in the release of Ach and stimulate cholinergic neurons. Morphine can inhibit the pain area of the cerebral cortex and has strong analgesic effect. It can inhibit the respiratory center and cough center and excite the smooth muscle of the bile duct, ureter, and bronchus, increasing its tension. After entering the body, morphine can be distributed in the hair of different parts of the body and can remain in the hair for a certain time, up to more than 10 weeks.

### 2.2. The Mechanism of Penehyclidine Hydrochloride against Morphine

PHC showed the same inhibitory effect as scopolamine on the withdrawal symptoms of morphine-dependent rats. PHC inhibits CPP in morphine-dependent rats, leading to central M receptor block, and can damage the memory of morphine-dependent rats and stimulate and affect the formation of CPP in rats. Many studies have shown that acetylcholine is mainly involved in the formation of M receptor-mediated morphine dependence and tolerance. M receptor agonists or central cholinergic drugs can cause opioid withdrawal symptoms. M receptor antagonists can reduce the withdrawal symptoms caused by naloxone. All these indicate that Ach and its M receptor are involved in the formation of morphine dependence.

### 2.3. Central Mechanisms Related to Addiction Mechanisms

#### 2.3.1. Midbrain-Limbic System Brain Area

The parietal system includes the subcortical nucleus and the parietal lobe. The marginal leaves are the medial hemisphere, the pear-shaped pod, the compartment, the hippocampus structure, and the cortex that surrounds the body's potassium in a convex circle. At present, the parietal system is divided into three parts: the ventral part of the frontal lobe, the structure of the medial frontal-parietal system, and the medial frontal gyrus. Various addictive drugs directly or indirectly act on the midbrain-parietal system, changing the neurotransmitters and receptors in various structures of the midbrain-limbic system, leading to addictive behaviors.

#### 2.3.2. Hippocampus

The hippocampus belongs to the ancient cortex, and its structure is located inside the hemisphere. Studies have shown that the hippocampus function is not only related to recent memory but also related to emotional control or emotional response that may affect the upward stimulus system of the brainstem network structure. Studies have shown that the hippocampus is a related area of the brain that plays an important role in the process of learning and memory and it participates in enhancing drug addiction. There are more and more studies on the relationship between the hippocampus and morphine dependence. Studies have shown that the AMPA receptor (*α*-amino-3-hydroxy-5-methyl-4-isoxazole propionic acid), N-methyl-D-aspartate receptor (NMDA), Ca2^∗^/CaM-dependent protein kinase II extracellular signal kinase (ERK), and hippocampal plastic molecules are involved in the formation of opioid dependence. The hippocampus plays an important role in consolidating short-term memory and transforming it into long-term memory. Protein inhibitor synthesis prevents the process of memory consolidation. In the process of memory consolidation, long-term enhancement plays an important role. Long-term enhancement, also known as long-term gain effect, is a lasting enhancement phenomenon in the signal transmission of two neurons, which can stimulate two neurons synchronously. This is one of the several phenomena related to synaptic plasticity—the ability of synapses to change intensity. Since memory is thought to be encoded by changes in synaptic strength, LTP is generally regarded as one of the main molecular mechanisms that form the basis of learning and memory.

## 3. Experimental Study on the Central Mechanism of Penehyclidine Hydrochloride against Relapse Behavior in Morphine-Dependent Rats

### 3.1. Experimental Materials

#### 3.1.1. Animals

56 purebred male Sprague-Dawley (SD) rats, weighing 160 ± 30 g, purchased from the Drug Safety Evaluation Center (GLP) of the City University of Chinese Medicine, were used; the number of animal quality certifications is as follows: SCXK (black). The feeding conditions are purebred laboratory, normal light, normal temperature control, room temperature control at 20°C~25°C, and relative humidity control at 50%~60%. The rats are kept in separate cages and can eat and drink freely. The rats were acclimatized to the environment for 1 week before the start of the experiment. The excretion of animals during the experiment meets the requirements of animal ethics.

#### 3.1.2. Experimental Setup

The Morris water maze (Smart3, 5, Shenzhen Reward Life Technology Co. Ltd) was used. The water maze is a large aquarium with a diameter of 120 cm and a height of 50 cm. The walls are uniformly black, divided into four areas I, II, II, and IV. The midpoint of each quadrant wall is the water inlet point, which is located at the center of quadrant II. Install a cylindrical transparent platform with a diameter of 12 cm and a height of 29 cm at a distance of 30 cm from the edge. The water tank was filled with 30 cm deep water, so the platform sank to 1 cm below the water surface. The water temperature is controlled at 25 ± 1°C. The screen system is located above the maze, and an automatic camera system is installed. Electronic balance (PL602-L): METTLER TOLEDO Instruments (Shanghai) Co., Ltd., Multifunctional high-speed centrifuge: Heraeus, Germany, refrigerator: Hefei refrigerator factory, 722 UV spectrophotometer: Beijing RiliM, microscope: OPTEC BK 5000, inverted fluorescence microscope: S70 LEICA DMIRB, image analysis system: Image-Pro Plus 6.0, microplate reader model: DENLEY DRAGON Wellscan MK 3, plate washer model: Wellwash 4MK2, digital display: PYX-DHS, Eddy current mixer model: XW-80A. Note that the Morris water maze is an experimental device that enables animals to swim and find a platform hidden in the water. It is mainly used to test the learning and memory ability of spatial position and direction of experimental animals.

### 3.2. Experimental Method

#### 3.2.1. Animal Grouping

The rats were randomly divided into the blank control group (k), PHC low-dose group (LP according to a body weight of 0.22 mg/kg), middle-dose group (MP according to a body weight of 0.55 mg/kg), high-dose group (HP according to a body weight of 1.38 mg/kg), and medicine group, with 40 rats in each group. Each group was randomly divided into 5 subgroups (*n* = 10): 4 h after administration, 7 h after administration, 13 h after administration, 25 h after administration (K48, LP48, MP48, and HP48), and 37 h after administration.

#### 3.2.2. Administration

Each rat was given intraperitoneal administration and immobilized. The needle was pierced into the skin of the lower abdomen near the white line and then pierced into the abdominal muscle at a 45° angle to the skin. Abdominal muscles and resistance disappear and enter the abdominal cavity. The dosage of the medicinal solution was 0.15 ml/10 g, and the control group received the same amount of normal saline. The rats were not allowed to eat or drink within 6 hours after administration. After six hours, they were free to eat and drink. Control is one of the means controlled by the experiment. The purpose is to eliminate the influence of irrelevant variables on the experimental results and enhance the credibility of the experimental results. In the control test, the experimental group and the control group are involved. As for which is the experimental group or the control group, the judgment basis is different in different control types.

### 3.3. Experimental Procedure

#### 3.3.1. Morris Water Maze Experiment (Conducted at 8 am)

Divide the experiment into two stages, between p11-p16 (stage i) and p18-p24 (stage ii). The content of the first stage mainly includes the experiment of directional navigation and the experiment of space detection. The experimental time of the navigation direction is generally 6 days, and the rats are trained 5 times a day. Each time a mouse is placed underwater at four fixed entrances facing the wall of the pool, allowing a search time of 65 seconds. Once found, it will stay on a platform for 15 seconds. If not, please guide the mouse to the platform and hold it tightly for 20 seconds. The downstream water flow sequence changes randomly every day. Record the incubation period of a mouse when it is on the stage [take the average of the incubation period of 5 measurements as the day The best escape time], the exercise strategy can generally be divided into four types: edge strategy, if the mouse needs to spend more than 71% of the time to get away from the circle, center on the area of the mouse's normal movement, run 70% of the length. The software system takes the movement of the mouse as a fringe strategy. Linear strategy, if the distance between all points on a rat track and the central axis does not exceed 10% of its radius, and the time to move around the central axis in a designated area should account for at least the amount of movement of the total central axis 71%, the movement with the time of moving around a water platform as the central axis is clearly defined as linearity, indicating that the rat gradually forms a cognitive reference in the maze. The trend is similar to the linear strategy, but the range of motion is within 50% of the radius. The mouse using this strategy is basically correct in determining the position and direction of the target, but the positioning accuracy is still insufficient. The above three are different; then, the system judgment is random.

#### 3.3.2. Immunohistochemical Detection of the Rat Brain Hippocampus

(*1) Preparation of Specimens*

The right brain tissue was washed with ordinary water, placed in a 50 ml centrifuge tube, and poured into 31 ml of neutral formaldehyde (55 m of 135% formaldehyde solution + 550 ml of distilled water to form 5% neutral formaldehyde). Correct fixation in 24 hours, Q8 hours inverted in the centrifuge tube. In order to quickly remove the forehead of the rat, the sample was rinsed under running water for 12 hours, referring to the George Paxinos gap to the limit. Use a graduated knife to cut 3 cm^∗^4 cm^∗^5 mm paper towels on the surface of the crown and mark them. Be careful not to pull the tissue. The remaining samples are placed in neutral formaldehyde solution for later use. Dehydration, transparency, embedding: the sample is placed in 80% alcohol for 2 hours-→90% alcohol soak for 12 hours → 95% alcohol soak for 1 hour → 100% alcohol for 40 minutes → 100% alcohol for 60 minutes → xylene I 15 minutes xylene II 30 minutes-→drying->add hard wax at 70°C, room temperature 33°C-→put the sample into the cooling section of the refrigerator: use a microtome to cut the sample into 6 *μ*m thickness→adhesive→dry with a hair dryer.

*(2) Mount the Slide, Observe the CA1 Area of the Hippocampus, Calculate the Number of GFAP Immune Cells in each of the Three Adjacent Fields of View, and Take the Average of the Three Fields of View. Count the Number of GFAP-Positive Cells*

### 3.4. Data Processing

1. In the statistical processing method of biochemical content determination, data are expressed as mean ± standard error. The average of the three samples before the administration was used as the baseline and set to 100%. The change every 20 minutes after dosing is expressed as a percentage of baseline. Perform statistical analysis on the data through iterative measurement analysis. Grouping is used as a between-group factor, and time points are used as a within-group factor. The difference between the two groups was analyzed by LSD. Use one-way analysis of variance to compare the differences between groups at each time point. In the real world, the data are generally incomplete and inconsistently dirty, which cannot be directly mined, or the mining results are not satisfactory. In order to improve the quality of data mining, data preprocessing technology is produced. There are many methods of data preprocessing: data cleaning, data integration, data transformation, data reduction, and so on. These data processing technologies are used before data mining, which greatly improves the quality of data mining patterns and reduces the time required for actual mining
2. Before measuring the correlation between variables and linear variables, the regression model must first be adapted to predict the average value of *θ* (direction linear correlation coefficient) when a specific *θ* or a specific random variable *X* = *x*. There are obvious differences between these two regression models, and the correlation coefficients are also very different

In the linear-directional model, when the value of *θ* is given by the measurement, the mean value of *X* is predicted and the model is

(1) $$\begin{array}{c} E\left(\left.X\right|\Theta =\theta \right)=a_{0}+b_{0}\cos\left(\theta -\theta_{0}\right). \end{array}$$

The above formula can be transformed into

(2) $$\begin{array}{c} E\left(\left.X\right|\Theta =\theta \right)=a_{0}+\text{a}\cos\theta +b\sin\theta . \end{array}$$

In the latter equation, for the linear regression of cos*θ* and sin*θ*, the regression coefficients can be calculated by traditional methods, so there is no need to further explain the relevant content of the regression model but it is very helpful to explain the relevant content of the regression model. The regression model prediction method is a prediction method based on the regression method of quantitatively studying the correlation between variables. The basic idea is through the sample information, analyze the overall correlation between the prediction object and relevant factors and set an appropriate mathematical model to express the types of this correlation. Then, using the sample information and parameter estimation method, a sample regression model reflecting the overall relationship between the prediction object and the main relevant factors is established. Carry out necessary inspection. Finally, according to the established and tested sample regression model, the future situation of the research object is predicted.

## 4. Analysis of Experimental Results

### 4.1. Morris Water Maze Experiment Results

#### 4.1.1. Exercise Strategy

The exercise strategy data of each group of mice obtained through the Morris water maze experiment are shown in Table 1.

It can be seen in Figure 1 that the four groups of rats used more effective straight line and tension strategies. The four groups had no significant difference in the use of edge strategy, trend strategy, and random strategy (*P* > 0.05). The linear search strategy of 4 groups was significantly smaller than that of 1 group, and the difference was significant (*P* < 0.05).

#### 4.1.2. New Object Recognition

The new object recognition data of each group of mice obtained through the Morris water maze experiment are shown in Table 2.

It can be seen in Figure 2 that the phase I (P21) preference index of the four groups of rats showed a downward trend and there was no significant difference between group 4 < group 3 < group 2 and group 1 (all *P* < 0.05), group 2 and group 1 > 0.05); the second stage (P34) preference index has no significant difference (*P* > 0.05).

### 4.2. Measurement Results of TchE Activity and Ach Level in the Hippocampus

The rat brain hippocampus was detected by immunohistochemistry, and the results of the determination of TchE activity and Ach level in the hippocampus are shown in Tables 3 and 4.

It can be seen in Figures 3 and 4 that 4 and 7 hours after administration, compared with the first group, the TchE activity of the second, third, and fourth groups increased and the Ach level decreased (*P* > 0.05). At 25 and 37 hours, the TchE activity and Ach level of the second group were not significantly different from those of the first group (*P* > 0.05); the first group was compared with the second and third groups of TchE, and the activities of the fourth and fourth groups were increased, and the level of acetylcholine (*P* < 0.05) was decreased. Compared with that of the third group, the TchE activity of the fourth group increased and the Ach level decreased and the difference was significant (*P* < 0.05). In nerve cells, acetylcholine is synthesized by choline and acetyl CoA under the catalysis of choline acetyltransferase. In animal cells, acetylcholine directly affects the permeability of membrane to ions on the one hand and affects the progress of various physiological processes through various second messengers on the other hand.

## 5. Conclusions

In this paper, the central mechanism of penehyclidine hydrochloride against the relapse behavior of morphine-dependent rats is studied. After analyzing the relevant theories, the experimental verification is carried out. The experimental results show that the four groups of experimental mice were tested in the Morris water maze experiment. Choosing a more effective straight line and tension strategy, after analyzing the hippocampus tissue, it is concluded that PHC can reduce the Ach level in the hippocampus of mice, which leads to memory impairment in mice.

## Figures and Tables

**Figure 1:** Exercise strategy experiment results.

**Figure 2:** New object recognition experiment results.

**Figure 3:** After administration TchE activity in all groups.

**Figure 4:** After administration Ach level in all groups.

**Table 1:** Exercise strategy experiment results.

	1	2	3	4
Fringe	11%	11%	10%	12%
Trend	31%	31%	33%	34%
Linear	40%	38%	37%	36%
Random	19%	21%	21%	23%

**Table 2:** New object recognition experiment results.

	Phase I preference index (%)	Phase II preference index (%)
1	63.68	69.68
2	62.36	71.94
3	56.08	70.56
4	51. 05	68.58

**Table 3:** After administration TchE activity in all groups.

	4 h	7 h	13 h	25 h	37 h
1	0.326	0.328	0.311	0.295	0.291
2	0.442	0.536	0.328	0.340	0.331
3	0.434	0.504	0.614	0.592	0.658
4	0.547	0.539	0.733	0.744	0.752

**Table 4:** After administration Ach level in all groups.

	4 h	7 h	13 h	25 h	37 h
1	0.316	0.286	0.311	0.295	0.291
2	0.472	0.506	0.318	0.320	0.311
3	0.494	0.492	0.604	0.593	0.645
4	0.507	0.489	0.723	0.794	0.812

## Data Availability

The data underlying the results presented in the study are available within the manuscript.
